RETRACTED

# Software Systems Security Vulnerabilities Management by Exploring the Capabilities of Language Models Using NLP

**DOI:** 10.1155/2021/8522839

**Published:** 2021-12-27

**Authors:** Raghavendra Rao Althar, Debabrata Samanta, Manjit Kaur, Abeer Ali Alnuaim, Nouf Aljaffan, Mohammad Aman Ullah

**Affiliations:** ^1^Data Science Department, CHRIST Deemed to Be University, Bangalore, Karnataka, India; ^2^QMS, First American India Private Ltd., Bangalore, Karnataka, India; ^3^Department of Computer Science, CHRIST Deemed to Be University, Bangalore, Karnataka, India; ^4^School of Electrical Engineering and Computer Science, Gwangju Institute of Science and Technology, Gwangju, Republic of Korea; ^5^Department of Computer Science and Engineering, College of Applied Studies and Community Services, King Saud University, P.O. Box 22459, Riyadh 11495, Saudi Arabia; ^6^Department of Computer Science and Engineering, International Islamic University Chittagong, Chittagong, Bangladesh

## Abstract

Security of the software system is a prime focus area for software development teams. This paper explores some data science methods to build a knowledge management system that can assist the software development team to ensure a secure software system is being developed. Various approaches in this context are explored using data of insurance domain-based software development. These approaches will facilitate an easy understanding of the practical challenges associated with actual-world implementation. This paper also discusses the capabilities of language modeling and its role in the knowledge system. The source code is modeled to build a deep software security analysis model. The proposed model can help software engineers build secure software by assessing the software security during software development time. Extensive experiments show that the proposed models can efficiently explore the software language modeling capabilities to classify software systems' security vulnerabilities.

## 1. Introduction

Software has become a core part of human life and plays a prominent role in day-to-day activities. With advances in technology, loopholes are also getting created at a rapid pace. Software development organizations consider the security of the software as a prominent part of their focus area for customers. However, there are extensive knowledge sources available across the industry within and outside the organization. Due to the continuously changing priorities of the organization, security knowledge takes a back seat. There is a need for devising a proper mechanism to assimilate all the knowledge prevalent in the industry and provide it to the software development team in a controlled way as and when they need it. It requires an intelligent way of putting the information together, learning from them continuously, and using the learnings in operations. There is a need for a smart knowledge management system for the security of the software systems. A smart knowledge management system will be the system that will have the capability to integrate the data from various sources. And this integrated source of required information is made available for the one interested at the right point of time in software development processes. The system will have to be fed in with the events from the outside organization and within the organization. All the data processed within the software development value stream will also be leveraged for this knowledge system. Customer conversations with the technology team will hold prominence as they may have the software system's explicit and implicit security needs. This paper is focusing on streamlining the software engineering process by leveraging the artificial intelligence approach. Security concerns of the software engineering processes are targeted. This focus area aligns with the journal's scope, as the journal intends to bridge the gap between engineering, artificial intelligence, and neuroscience.

RETRACTED

Leveraging the latest data science advancements for this problem area will bring efficiency in managing this domain. Most of the data will be a natural language, so NLP (natural language processing) approaches will be explored. Data related to a conversation with customer and software requirements management team is natural language data. Good practices documented in the security management platforms in the industry provide natural language inputs. Within the software development landscape, there are natural language data like security scan-related outcomes. These rich data forms make NLP a go-to framework for modeling. All these data sources have hidden patterns for the possible security flaws that would creep into the system. With some good language processing capabilities emerging in the field, their relevance has to be studied. The research area taken up involves building a comprehensive knowledge management system to facilitate secured software development. The system will be banking on the data sources from the industry, the company, and the data processed during conversations between customer and software development teams. The paper's focus is to explore some of the key constructs associated with this system envisioned.

Furthermore, the experiment is taken to the next level by exploring NNLM (neural network language model) and BERT (bidirectional encoder representations from transformers). NNLM is a neural network-based language model that focuses on learning the distributed representation from language. This focus helps reduce the complexity of modeling a language due to a large number of features. BERT is a specialized state-of-the-art model for language modeling. BERT is studied in different formats for data modeling. BERT as vectorizer, tokenizer, and other capabilities of BERT are explored. DCNN (deep convolutional neural network) is the following approach explored, followed by BERT's capability to set up a question answering system. Exploration is essential as the overall architecture of this knowledge management system provides the necessary knowledge to the software development team to be handy in this setup. TensorFlow and PyTorch implementation aspects are discussed, later moving on to the possibilities of learning from the source code that holds some core knowledge about the software systems. As a roundup, some of the research gaps and prospects are explored.

RETRACTED

The remaining paper is organized as follows. In Section 2, scope of ethe work is presented. In Section 3, the literature review is presented. Constructs of language models are discussed in Section 4. Data set considered for experiments is demonstrated in Section 5. The experimental setup, which considers various models, is presented in Section 6. Experiments exploration is presented in Section 7. BERT exploration is illustrated in Section 8. Key constructs of the security knowledge management system are elaborated in Section 9. The learning from source code is demonstrated in Section 10. The concluding remarks are given in Section 11.

## 2. Scope of Work

Real-world data consists of unbalanced data and unlabeled ones. Unbalanced data includes those data where a particular class of data is predominant over the others. Deep transfer learning plays a prominent in the space of NLP in these situations. Pretrained models have made the processing of these problems much more efficient and effective. In this study, we explored the security landscape in software development to ease the life of software developers and other team members by providing security-critical information.

## 3. Literature Review

### 3.1. Text Analysis

In [1], the effort involved in labeling the text data was reduced using supervised learning. Kohonen self-organizing map (SOM) was employed for labeling the data. Accuracy of classification was validated using a decision tree, Naive Bayes, support vector machine, and classification and regression tree algorithms. In [2], the text classification approaches were surveyed for unstructured mining data. The strengths, weaknesses, opportunities, and threats (SWOT) were explored to know the trend of their usage. Software security vulnerabilities are loopholes in the software system that can compromise the data within the system. Some of the examples can be missing authentication for an important function and missing data encryption.

RETRACTED

In [3], text data mining was done using the back and forth matching (BFM) algorithm to make the pattern matching a faster process. In [4], the optimized named entity recognition (NER) approaches were explored for expectation-maximization with semisupervised learning approaches. In [5], authors identified different requirements for linguistic analysis such as linguistic rules, incorporation of NLP, and so on. In [6], authors consider the need of experimenting with NLP or machine learning or other text analysis approaches as a separate focus area, beyond their attempt to run a combination of these techniques. Formalizing the structure of the software requirements can help standardize the conditions outlined for the organization to ensure that security-related requirements get their focus right at the beginning of the software development, which can potentially reduce the cost and effort.

### 3.2. Software Processes Analysis

Technical debt is an essential consideration in this paper. Some studies identified the influencing factors for technical debt in software systems. These are gathered during the software development process when there is an attempt to balance the customer's strategic and short-term needs.

The anomaly detection method was introduced in [7], which leveraged the optimized mechanism of routing the raw features of the problem area inside a Boltzman machine algorithm. In [8], a software fault detection and correction modeling framework was proposed in software testing. In [9], a software effort estimation approach was proposed for the agile software development model. Artificial neural network feedforward, backpropagation neural network, and Elman neural network were employed. In [10], a variety of nonfunctional requirements were considered for modeling and to set up an appropriate pipeline to update the criteria and send it across to the next phase [11].

In [12], the security controls were identified using automated decision support. These controls can be relevant to any specific system. In [13], a security requirement elicitation approach based on problem frames was proposed. It considered the incorporation of security into the software development process at an early stage. It helps the developers gather information regarding security requirements in an efficient way. A security catalog was prepared to identify the security requirements, and threats were accessed using abuse frames.

RETRACTED

In [14], machine learning techniques were assessed to identify the software requirements for stack overflow. It showed that latent Dirichlet allocation (LDA) was used widely to identify the software requirements. In [15], a tool was devised to discover the vulnerabilities based on the features of software components. The software component features represented the domain knowledge in other software development domains. Since the approach prescribed targets to predict the vulnerabilities in a new component, there is potential to leverage the history of the vulnerabilities for these software components in the production. There is also the potential of taking these solutions and integrating them into the development environment for ease of usage to software developers. The overall emphasis is to make software systems secure right from their inception. It can cut down on the need for the significant investment made by companies for the security of the software.

### 3.3. Machine Learning

The fixing time of a security issue within the project significantly impacts the overall development process. Therefore, it is essential to fix the issue within a timeline. In [16], machine learning models were used to predict the fixing time. In [17], long short-term memory (LSTM) technique was used to classify the spam. This technique can learn abstract features automatically. In this, the text was changed into semantic word vectors using ConceptNet and WordNet. After that, spam was detected using LSTM from the data. In [18], the accuracy of the K-nearest neighbor (K-NN) algorithm was improved in classification tasks. However, it takes a longer time in large data sets but provides significant accuracy as compared to others. In [19], the security requirements mentioned in the software requirement specification document were mined. These requirements were classified as data integrity, cryptography, access control, and authentication using a J48 decision tree. After that, prediction models were developed for each security requirement. The pretrained models can also identify the wrongly classified requirements in the document to provide better insight to the requirements engineer. The further refinement will give users the classified information on requirements and explain why a particular classification was chosen. It is a challenging issue with a neural network that needs a better approach to make an interpretable model.

## 4. Constructs of Language Models

It is essential to understand the construct of the language model that effectively applies to solve the problems associated with software security issues. Problem related to software security can be solved by leveraging the natural language data that is available across companies and industries. Effective language modeling capabilities can help derive the information hidden in these data. Further from this, security-related information can be leveraged by the software development team as and when they need it. Language models are the basis of the models that used in this paper. Language models find their roots in the N-gram modeling approaches. N-gram modeling uses the thought process of assessing the probability of a given the word using its history [20]. For example, the probability of the next word in the phrase “Jack and Jill went up the” to be “hill.”

(1) $$\begin{array}{c} P\left(\text{hill}|\text{Jack and Jill went up the}\right). \end{array}$$

One of the approaches used to compute this probability is relative frequency. By taking the corpus of language as a base, how often the word “hill” follows the phrase can be calculated as follows:

(2) $$\begin{array}{c} P\left(\text{hill}|\text{Jack and Jill went up the}\right)=\frac{C\left(\text{Jack and Jill went up the hill}\right)}{C\left(\text{Jack and Jill went up the}\right)}, \end{array}$$

where *C* represents the count of occurrence of the phrase. The chain rule of probability is applied to words to obtain the following expression:

(3) $$\begin{array}{c} P\left(W_{1:n}\right)=P\left(w_{1}\right)P\left(w_{2}|w_{1}\right)P\left(w_{3}|w_{1:2}\right)\ldots P\left(w_{n}|w_{1:n-1}\right)\\ =\prod_{k=1}^{n}P\left(w_{k}|w_{1:k-1}\right), \end{array}$$

where *w* denotes the word, *n* represents a word count, and *k* represents the length of the sequence. To simplify the complexity of dependencies on the word, Markov assumptions are employed [21]. This assumption emphasizes that the probability of future prediction can be done with just a few instances from history. In the case of N-gram, it will be enough to look at *n* − 1 previous words. Maximum likelihood estimation is used for calculating the probabilities of N-grams as follows:

(4) $$\begin{array}{c} P\left(w_{n}|wn-1\right)=\frac{c\left(w_{n-1}w_{n}\right)}{w_{n-1}}. \end{array}$$

RETRACTED

## 5. Data

This paper takes the data set from a software development team that works on an insurance domain project. All the customer requirement-related data and internal software development process-related data such as test cases and defects are taken and labeled as security- and nonsecurity-related data classes. Thus, the data set contains the text and corresponding labels. Data set contains natural language data obtained from customer requirements specifications, test cases, defects, and other software development work maintained by the software development team. Data set is divided into training, testing, and validation in the ratio of 50%, 40%, and 10%, respectively. The software development requirements management experts labeled the data that are associated with customer requirements. Software development technical leads are involved in labeling the data associated with software development work, such as defects and test cases. Data set is randomly split into training, testing, and validation using the train-test split library of python. We have considered various fractions of training and testing data. It is found that when the training data set fraction is 50%, then the model does not suffer from over- and underfitting issues. There are 31,342 data points, with 3,082 security-related ones and 28,260 nonsecurity-related data points. Therefore, data augmentation techniques such as back translation [22] and easy data augmentation [23] are used to balance the data set. Since some of the deep learning approaches are explored, basic text cleaning methods are only applied. NLTK is used for text cleaning purposes.

Preprocessing of the data includes tokenization of the text to create a vocabulary. Text is first converted to sequence of words and then converted to sequence of numeric IDs. Tokenization of the text involves the conversion of the text into numerical representation so that these representations can be passed into machine learning or deep learning models for modeling purposes. Text sequence padding is also done to normalize the text sequence length. Data are represented as a vector sequence for further modeling.

## 6. Experiments Set Up

In the first experiment, CNN is explored in text classification [24–26].  Algorithm 1 demonstrates the various steps involved in text classification using CNN. Firstly, text data is tokenized using the TensorFlow Keras preprocessor. Text sequences are transformed into a sequence of numeric IDs. So there will be three sets of text sequences for training, testing, and validation.

Sentence length distribution is visualized to check the length distribution. The maximum sequence length for padding can be kept at 250, as most of the long sequences fall within a sequence length of 250. TensorFlow Keras preprocessor is used to create text sequences of 250 lengths for all three sets of the data set.

In the next stage, a pretraining-based fastText embedding matrix is explored [27–29]. fastText is an open-source lightweight library that helps learn the text representation in the language models. fastText is configured as a matrix of the data that it has already learned during its pretraining, in the form of embeddings of the numerical representation. The pretrained model, “wiki-news-300d-1M-subword.vec.zip,” provides 1 million word trained vectors from the information of Wikipedia. fastText works are similar to word2vec, where each word is considered for its bag of character-based N-grams. Pretrained word embedding architecture is built in a standard way. An embedding size of 300 is chosen for this pretrained model that is constructed on 300 dimensions. TensorFlow Keras-based CNN model architecture is built (see Algorithm 1). Three sets of Conv1D and max-pooling layers are built using 256, 128, and 64 filters in each of the Conv1D layers and a pool size of 5 for the max-pooling layer. The activation function applied is “ReLU” (rectified linear unit) [30, 31]. The architecture has three sets of dense and dropout layers, with a dropout set at 25%. Binary cross-entropy loss [32, 33] and Adam optimizer [34] are configured for model compilation. Model architecture is run on the training data set. Though the model is configured to be run for epochs count of 100 and batch size of 128, with early stopping, the model reached optimum accuracy on 7th epoch, with validation accuracy of 95.95%. Model performance is evaluated on the test data set; it showed an accuracy of 71.89%. A weighted average of precision is 0.88; recall is 0.72; and F1-score is 0.77. Without much fine-tunning of the parameters, the model would provide an accuracy of 71.89%. Therefore, these architectures can be further fine-tuned for the insurance data to achieve better accuracy.

RETRACTED

The experiment is further topped up with a bidirectional LSTM and attention layer (see Algorithm 2). The embedding layer is retained with a pretrained FastText model. Tokenization, vectorization, and padding are conducted similarly to the earlier part of the experiment. The output from the last layer of the long short-term memory gated recurrent unit (LSTM GRU) is fed into the global attention layer sequence.

(5) $$\begin{array}{c} e_{t}=a\left(h_{t}\right)=\tanh\left(Wh_{t}+b\right), \end{array}$$

(6) $$\begin{array}{c} \alpha_{t}=\text{softmax}\left(e_{t}\right)=\frac{\exp\left(e_{t}\right)}{\sum_{k=1}^{T}\exp\left(e_{k}\right)}, \end{array}$$

(7) $$\begin{array}{c} c=\sum_{t=1}^{T}\alpha_{t}h_{t}. \end{array}$$

Vectors from the hidden sequence are passed on to a learning function (*h*_*t*_), including a product vector. *c* is the final context vector, and *T* is the total time steps for the input sequence. Attention layer architecture is based on the TensorFlow Keras attention mechanism for temporal data and masking. TensorFlow is a machine learning library, and Keras is the high-level API of TensorFlow. Attention mechanism is the cutting-edge approach for leveraging the learning from essential parts of the language rather than trying to learn everything. TensorFlow and Keras's attention mechanism provides tool for implementing this capability in the model. Constructs used in this experiment are taken from [35]. FastText-based embedding is built as in the first part of the experiment. Core model architecture is built with LSTM to form the sequential models. LSTM is better than RNN in remembering the long sequence of data. LSTM manages input at the current time step, with the output of the previous LSTM unit and memory of cell state in the previous unit.

RETRACTED

Bidirectional LSTMs help feed both forward and backward sequences of the content. The output provided by each of these is combined at every time step. By considering the past and future sequences, a better context of the text is retained. The architecture encompasses embedding as input, bidirectional LSTM GRU with 256 units, attention layer, and three sets of dense and dropout layers (see Algorithm 2). Two hundred and fifty-six units for thick layer and 0.25 dropout rate are also used alternatively. “Relu” is the activation function used for intermediate layers; in the final layer, “sigmoid” is used. Binary cross-entropy loss and “Adam” optimizer are also considered. Model is trained with an early stop mechanism for 100 epochs feeding in training and validation. A batch size of 128 is retained; best results are reached at the 6^th^ epoch, with a validation accuracy of 98.69%. The model achieves an accuracy of 84.33% with weighted average precision of 0.91, recall of 0.84, and F1-score of 0.87.

In the next phase of the experiment, Google's Universal Sentence Encoder (USE) is explored. It can encode high-dimensional vectors with varying lengths into a standard size.  Figure 1 shows the working of sentence encoding.

In this experiment, USE is implemented on TensorFlow 1.0. USE model is loaded from the TensorFlow hub [36]. The USE-based embedding layer is constructed and fed into the model architecture with two dense and dropout layers (see Algorithm 3). The dense layer has 256 units and a ReLU activation layer, with a dropout value of 0.25. The sigmoid activation function is used to classify the results. Binary cross-entropy and Adam optimizers are also used. Model training is implemented by considering the early stopping. It achieves an optimal validation accuracy of 97.32% in the first epoch. It has performed an average accuracy of 92.61%, with average recall, precision, and F1-score as 93.0%, 95.0%, and 93.0%, respectively.

## 7. Experiments Exploration

Software requirements modeling is one of the prominent parts of this work. Most of the time, the focus is on software correctness in the development that can lead to performance issues later in the development process. In [37], a comprehensive study of all the work done towards modeling the performance of the software across the software development lifecycle is presented. In [16], the factors that impact the time for fixing security issues with linear regression methods are assessed.

RETRACTED

The focus of [38] is to look at machine learning applications for software vulnerabilities management and various data mining approaches. Vulnerabilities discovery models with software metrics, vulnerable code pattern identification, and anomaly detection methods are explored. In [39], the focus is given on technical debt being used as a base for security issues modeling with machine learning. In [40], a focus is presented on applying a set of hybrid codes covering static and dynamic variables that characterize input validation and patterns of input sanitization code, and these are expected to be prominent indicators of vulnerabilities in web applications. There is a good complement between static and dynamic program analyses; both techniques extract the proposed variables in a scalable and accurate method.

Building on the base constructs experimented with within the previous section, this section explores more advanced architectures. NNLM is explored in this section. Sentence encoding is experimented with NNLM, which also provides fixed-length vectors for the documents. The exact format of data processing is continued in this section as well. NNLM model is fetched from the TensorFlow hub from https://tfhub.dev/google/tf2-preview/nnlm-en-dim128/1 [41]. Keras layer is built from the hub with an output shape of 128. Model architecture is built with Keras layers from TensorFlow that will have pairs of dense and dropout layers. The dense layer will have 128 units and “ReLU” activation; The value for the “dropout” is chosen to be 0.15, with loss function of “binary cross-entropy”; and ‘adagrad' optimizer is determined (see Algorithm 4). Model is fit with the train data for 100 epochs and a batch size of 128. At the end of 100 epochs, the model reached a validation accuracy of 90.17%. The model demonstrated 90.16% accuracy on test data with an average precision rate of 0.81, recall of 0.9, and F1-score of 0.86.

BERT is explored in the next part of the experiment. Simple BERT architecture is shown in Figure 2. BERT undergoes semisupervised learning on a large amount of online data such as Wikipedia. Language understanding capabilities are inherent in these pretrained models that can be leveraged to many of the tasks associated with language processing. These pretrained models can be refined to different data sets with less effort to use their capability concerning the specific domain of application. BERT expects the text content to be tokenized, and in lowercase, Hugging Face's https://huggingface.co/ [42].

RETRACTED

BERTTokenizer, which is part of transformers, is used. The word piece tokenizer approach segments the words into a subword level like any other NLP (natural language processing) task. The tokenizer is formed with the pretrained model, “bert-base-uncased.” Data used for this experiment need to be preprocessed with an approach similar to that of the original method used in the BERT pretrained model. Pre-processing includes, the conversion of data in to lower case, tokenization, breaking of word pieces, word to index mapping using BERT vocabulary, adding the seperator and end of sequence tokens, and finally appending, ‘mask' and ‘segment' tokens.

The model architecture here consists of the BERT that helps process the input data of text based on its prelearned language capability; on top of this, a feed-forward neural network with softmax is built for customized classification tasks. Models layers are made with TensorFlow Keras layers. A maximum sequence length of 250 was selected for the data used in this experiment, as most of the sentences fall within the range of 250 lengths of words. Input ID, mask, and segment are created with the hidden state made from the pretrained model “bert-base-uncased.” The further part of architecture will have dense and dropout layers of two, each alternating, followed by a dense output layer. Two hundred fifty-six units are used for dense layers, and a 0.25 dropout rate is considered. The “ReLU” activation layer is used in dense layers with “sigmoid” activation for the dense output layer. For a model compilation, Adam optimizer is used with a learning rate value 2*e* − 5 and 1*e* − 8 epsilon value, and binary cross-entropy loss and accuracy metrics are used.

The utility function that is created for converting the text input data to BERT features is used. The same training set used until this point is used here. To recap, this data is a customer requirement in an insurance domain, and test cases and defects data were created as part of software development operations on this insurance company. Data is labeled as security and nonsecurity data based on expert input. Data is prepared in a similar way to the earlier part of the experiments. Training data is converted to training feature IDs, training feature masks, and training feature segments using the BERT tokenizer constructed earlier. Now the built model is trained using the training and validation part of data passing in the IDs, masks, and segments. Three epochs and a batch size of thirteen are used with early stopping (see Algorithm 5). The model reached a validation accuracy of 99.11% within the second epoch. The refined model is stored for further usage. Test data is also processed similarly, and predictions are run on the test data. It gave an accuracy of 91.3%, average precision of 0.92, recall of 0.91, and F1-score of 0.88. Since the current focus is to build a pipeline of the knowledge management system for software vulnerabilities management, these experiments are not explored further to make it more customized to the insurance company data targeted here.

RETRACTED

Though pretrained models provided ease of modeling with no need to train from scratch, they ended up being of massive size. To tackle this, distilBERT will be explored next. DistilBERT compresses the BERT with the knowledge distillation technique. The distillation technique is a way of reducing the complexity of the BERT architecture to make it concise and small during the pretraining phase. During the distillation, 40% of the size is reduced, retaining 97% of its language understanding and making it 60% faster than BERT. The teacher-student training approach is used where the student is trained to replicate the model output that of the teacher. Hugging Face uses KL-divergence loss to train distilBERT. The approach reduced the number of parameters to almost half compared to BERT retaining the performance. BERT tokenization is conducted similar to the experiment's last part; data preparation and model architecture setup are also the same. Sixty-six million parameters are generated in this case, unlike BERT, which had 109 million parameters. Input features of training and validation set of data are also prepared similar to the last part; tokenizer used is “distilbert-base-uncased.” In the case of distilBERT, three epochs are run with a batch size of 20 and an early stopping mechanism (see Algorithm 6). The model reached a validation accuracy of 99.07% at the second epoch. The test data model demonstrated 94.77% accuracy, average precision of 0.95, recall of 0.95, and F1-score of 0.94.

With these basic building blocks, the AI-based knowledge management system for software security vulnerabilities can be conceptualized. The system will have three prominent parts to it. Software security model architecture is shown in Figure 3. Customer conversation modeling will take in all the content generated as part of the conversation with the customer and use it to learn the security needs for software. The second part will be industry landscape modeling that will depend upon all the knowledge sources in the industry and leverage the same to understand security from an industry expert's point of view. In the third part, software landscape modeling, all the information within software development processes is leveraged to build security knowledge for the software development team. Exploration done so far will help construct the customer landscape and industry landscape modeling.

RETRACTED

Deep transfer learning constructs have been explored in the experiment so far that can help build this knowledge system for the insurance-based company's software development team. Pretrained word embeddings of deep learning models are explored, covering FastText with CNNs or bidirectional LSTMs with attention layer, universal embeddings with sentence encoders, and neural network language model. Transformers are explored, covering BERT and DistilBERT. TensorFlow 2.0 is used as a base to leverage its capabilities.

The attention mechanism is an interesting thought process and discussed in [16, 43]. The author calls the attention they have used in their architecture “scaled dot-product attention.”

(8) $$\begin{array}{c} \text{Attention}\left(Q,K,V\right)=\text{softmax}\left(\frac{{\text{QK}}^{T}}{\sqrt{d_{k}}}\right)V, \end{array}$$

where “*Q*” stands for queries, “*K*” stands for keys, and “*V*” stands for values. Attention function is specialized with mapping queries to a set of key-value pairs, further to an output. All the entities query, key, values, and output are vectors. Input encompasses queries and *d*_*k*_, which are keys of dimension, and *d*_*v*_, which are the dimension values. Authors also have explored the multihead attention mechanism as follows:

(9) $$\begin{array}{c} \text{Multihead}\left(Q,K,V\right)=\text{Concat}\left({\text{head}}_{1},\ldots {\text{head}}_{h}\right)W^{o}, \end{array}$$

where head_*i*_=Attention(*QW*_*i*_*Q*, *KW*_*i*_*k*, *VW*_*i*_*v*).

Multihead attention facilitates the model to access information jointly from a variety of representations. “*W*” here is the parameter matrices; “*W*^*O*^” represents the parameter matrix for the output; and “head” is an attention head. The author also uses a position-wise feedforward network in their architecture. This network is used in encoder and decoder layers that are applied to each position separately and identically.

(10) $$\begin{array}{c} \text{FFN}\left(x\right)=\max\left(0,xW_{1}+b_{1}\right)W_{2}+b_{2}, \end{array}$$

where “FFN” is feedforward network, “*W*” stands for weight, bias is given by “*b*,” and “*x*” is the input.

The next phase of the experiment industry landscape and customer landscape can be modeled by building the following pipeline. Any events about the software processes that include security and nonsecurity will feed into this knowledge system; the first level of the task would be to screen the relevant events for the software teams to understand the need for software security. All the events that are not associated with security have to be removed. The next part of the pipeline should categorize the events further into security-related events and are closely associated with the insurance domain, which is the focus domain of this research. As the system is in the initial stage of development, security experts can be involved in screening the outputs generated by the model to act as an input for the model to calibrate itself.

RETRACTED

## 8. BERT Exploration

In [44], researchers have shown that sentimental analysis of software artifacts can improve various software engineering activities. BERT has been leveraged for language modeling natural language text in Stack Overflow posts, subjected to sentiment analysis. In the view of leveraging on the wealth of knowledge hidden in the open-source software ecosystem, authors in [45] have proposed software entity recognition methods based on BERT word embedding. In [46], the author proposes automatic text classification based on BERT to develop an environment for the internet of things. The approach used here uses text-to-dynamic character level embedding with BERT. Furthermore, Bi-LSTM and CNN output features are utilized to leverage the CNN for local feature extraction and bi-LSTM for its capability on memory to link back the extracted feature.

In [47], the author focuses on utilizing BERT's self-attention mechanism for bidirectional context representation for predicting the resolution time of the bugs, which can contribute towards a better estimation of the software maintenance effort and cost.

BERT provides capabilities such as tokenizer for data preprocessing, creating word embedding, and constructing the question answering system. These parts have to be validated with the data from the insurance domain where the knowledge management system is built. BERT is the latest specialized approach; leveraging its capabilities will help exceed other methods for the targeted use cases in this space. As per the approach followed in earlier sections, the experiment will be built step by step to explore each capability of BERT. In the first part, the BERT tokenizer's data processing capability has been experimented. TensorFlow 2.0 is leveraged here as well. The training data set composed in previous sections of the experiment will be used in this set of experiments. Data will have text derived from customer requirements, test case descriptions, and defect descriptions for insurance domain-related software development processes. The text would have security- and nonsecurity-related content; the other column is a label that classifies security and nonsecurity classes of the text by the experts. Security-related contents are those where information related to software security is available. This security-related information will help understand the security controls that are needed in the software systems. Nonsecurity-related content is the rest of the information related to software system development. Text preprocessing is done to remove any nonalphanumeric content, “https://” from any URLs (Uniform Resource Locator), and punctuations and white spaces, if any. BERT layer has to be created so that metadata associated with the same can be assessed; vocabulary size is metadata. The tokenizer is designed with features of a vocabulary file and lower casing. Vocabulary file is derived from BERT layer that is constructed from Keras layer from TensorFlow hub. The text embedding feature used is “bert_en_uncased_L-12_H-768_A-12” [48], with a trainable parameter set to “false” as the feature will be used as is without further training it for this experiment sake. The tokenizer is used to convert tokens to IDs bypassing the sentences of the cleaned data into the same.

RETRACTED

Further data set creation will involve adding padded batches of sentences; each batch of the sentence is padded independently. Padding helps optimize the padding tokens. Their length sorts sentences, and then padding is applied and then shuffled. Data set are transformed as tensors using the “from_generator” method of TensorFlow (tf_data.Dataset). A batch size of 32 is chosen for performing padding. Model building involves DCNN with the following architecture.  Table 1 shows the training specification of DCNN architecture.

DCNN model construct is expressed in Table 2. The further architecture will have layers built as follows.

All the layers formed in Table 2 are merged by passing in the training data. DCNN is fit with the training data. Test data produces an accuracy of 97.44%. DCNN model can be used to pass in the text and predict whether the text is security related or nonsecurity related, with a confidence level on the scale of 0 to 1 (see Algorithm 7).

The second part of this entire exploration approach would remain the same except for the additional step of creating word embeddings. Embedding creation includes the creation of IDs, masks, and segments. Ids are created by using the “convert_tokens_to_ids” function from the tokenizer. Masks are created on tokens using NumPy by padding to tokens, and segments are created appending the tokens into segments. An accuracy of 99.58% was the result with the BERT tokenizer and embedding being applied.

RETRACTED

In the third part, architecture is refined to build a question answering module using BERT. Some of the libraries used for this experiment are as follows. BERT question answering system library specifications is presented in Table 3.

The SQuAD (Stanford Question Answering Dataset) is a well-known data set to explore question answering systems. Input metadata creation is the first step, which takes training data in JSON (JavaScript Object Notation) file and vocabulary file as input. Training data consists of a paragraph of information, which provides context, a question from that text, and answers for those questions. TensorFlow record is created from these files. The training data set is created using the “create_squad_dataset” library, passing the TensorFlow record of the data produced. “BertSquadLayer” is constructed with TensorFlow Keras dense layers. The complete model of BERT will have a class of “BERTSquad” that will take in the BERT layer from Keras layer of hub (https://tfhub.dev/tensorflow/Bert_en_uncased_L-12_H-768_A-12/1). The trainable parameter is kept as “true.” BERT application function of this class will take in input word IDs, input masks, and input type IDs. As part of the training phase following configuration is set.  Table 4 shows BERT question answering system training phase specifications.

These are computationally intensive experiments; parameters are optimized based on the need of these experiments. Once the pipeline of this knowledge management system is organized, it can be further customized to improve effectiveness. The training data set is also made lighter to facilitate an easy start for the experiment. Optimizer is created using the function “create_optimizer,” and SQuAD loss function is created to compute loss. BERT SQuAD model is compiled passing in optimizer and SQuAD loss function. Training is conducted passing in training data sets in batches as inputs and targets. BERT SQuAD layer and loss function is passed in, and gradients are applied on optimizer for training purposes. At the end of one epoch of training, training loss was reduced from 5.94 to 2.50. Next is the evaluation phase, where the development data set is used. Evaluation examples are created using the “read_squad_examples” library. TensorFlow record format of this evaluation data set is generated. BERT tokenizer that was created earlier is used. The function is created to add features into the evaluation feature list that is created (see Algorithm 8). Once the evaluation feature is created, the TensorFlow record is generated for the same. Then SQuAD is created from this evaluation data set. Thereafter, prediction is utilized to build the dictionary-like collection. The “NamedTuple” function of the “collections” library is used to create a dictionary-like collection. It will generate batched output in a timely way. Collection, evaluation examples, and evaluation features are passed into the “write_prediction” function of “official.nlp.data.squad_lib,” which generates prediction output files.

RETRACTED

The evaluation script has a function for normalizing the answers, generating an F1-score, defining the exact match score, comparing the results with ground truth, and evaluating the data set with the predicted values. The evaluation script must be run with the development data by passing in predictions generated in previous steps. Step here produces a result with an F1-score of 77.26 and an exact match of 66.91%. The experiment was conducted with limited resources to understand the approach. Once the construct of the pipeline is worked out, these approaches can be further refined and customized to target domain data that is software development practices of the insurance domain.

Based on the comparative analysis, Table 5 provides the comparison of the accuracy of the models. Table 5 also explains the key processes involved in the modeling, which provides information about the complexity of the approaches. Now, this setup can be utilized to predict any of our data. Question and context text must be concatenated with a separator token after tokenization like it was done for training content. Utilities required for this phase of prediction are the BERT layer from the Keras layer of the hub, which takes in the pretrained BERT model like in earlier phases. A comparison of all the experiments is provided in Table 5. Vocabulary file is generated from this BERT layer, including the lower casing function. Both vocabulary file and lower casing function are passed into “FullTokenizer” to generate tokenizers. Other utilities include white space recognizer, text to words converter, tokenizing each word, and keeping track of the tokens and words. Processing is continued with creation of IDs, masking, and segment creation from tokens, and finally a function is created to take a question and context as input, and return a dictionary with three elements as expected by the model. Expected output are context words, correspondence between context tokens to context word IDs, and length of the question tokens. Answers can now be predicted by passing in question and context to create an input dictionary run on BERT SQuAD trained earlier. Some more refinement can be done to organize the interpretation for the reading answers as output for the input provided in context and question. The model was used to pass in the context and question related to software applications security from the target domain, and it produced the answers for the given context.

RETRACTED

Question answering systems can play a handy role in the intended knowledge management system for software security in the insurance domain, the primary focus area.

CNN is one of the prominent areas of exploration in the domain explored in this paper. Some of the exciting work done with CNN is as follows. Exploration in [49] and [50] aims at devising an improvised CNN-based approach to improve the bug localization task in software engineering. In [49, 51], a bidirectional LSTM algorithm is proposed based on CNN and independent RNN for malicious web page identification. Word2vec is used for training URL word vector feature for modeling. Input sequence illustration in BERT represents in Figure 4.

Attention models are another critical component explored in this paper. Attention layers are techniques used in a neural network for processing the input, which facilitates the process of focusing on a specific aspect of complex information. In the work of Software System Security Vulnerabilities Management, modeling of customer conversation, industry knowledge bases, and knowledge gathered in software development processes are done. Since the focus is on the security dimension of the content, attention models will help build the required focus around security. Some of the other interesting results using attention models are as follows. The inability of the software defect prediction at the granular level of code hinders the possibility of providing detailed information to developers. In [51], the ensemble learning techniques and attention mechanism is utilized to provide comprehensive information to developers pointing at the suspect line of code and method-level defect prediction. The lack of focus on nonfunctional requirements like usability and security is handled ad hoc and results in cost. In [52], modeling of nonfunctional requirements across the software product life cycle is explored. Pseudocode generation is one of the essential aspects of software engineering, as it involves a lot of effort. In [53], there is an effort to treat pseudocode generation tasks as a language translation task that involves programming language translation to natural language description using the neural machine translation model and the attention seq2seq model. Bag of words with Naive Bayes approach shows the accuracy of 90%, precision of 77.7%, and recall of 93%. Classification of unsupervised learning approach shows the accuracy of 73%, precision of 69.3%, and recall of 77.7%. Table 5 shows a series of experiments conducted in this work that shows improved performance on security issues classification as the approach was tuned for data from the insurance domain. It started with accuracy of 71.89%, with CNN and FastText embedding. Performance went up to 84.33% with bi-directional LSTM and FastText embedding. USE model made up to the accuracy of 92.61%; NNLM model made up to the accuracy of 90.16%; and BERT model would further refine the accuracy up to 97.44%. Experiments are started with conventional CNN with pretrained FastText embeddings. Pretrained FastText embeddings are further combined with bidirectional LSTMs and attention layers. Bidirectional LSTMs provide the ability to read the inputs from both directions and enhance learning. USE approach provides the ability to encode texts of any length in higher dimensions vector and is useful to try. NNLM model provides the ability to encode the sentence with a fixed length of vectors with pretrained layers for predicting the next word. BERT and DistilBERT are tried at the end, as they are the cutting-edge approaches and provide the ability to fine-tune the pretrained model to suit the targeted domain data. DistilBERT also has played a key role in reducing the size of pretrained models. The system proposed in this work focus on effectively handling security aspects in software development processes. The central theme of this exploration is modeling the data from customer conversation, information on public websites from the organization that works on educating the industry on security vulnerabilities, and data internal to software development processes. Most of this information is in natural language data, so it is beneficial to explore NLP-related approaches to tackle the problem. With the latest developments in the NLP space, some of the advancements around language models fit well to solve some of the areas targeted in this work. Advanced NLP will help pool all the unstructured data in and around software development and learn patterns from them. This aspect can be leveraged to solve some of the challenges software development processes face around the quality of work, productivity, and process maturity. In the further set of experiments, a 95% confidence interval will be considered for accuracy, F1-score, recall, and precision. This set of experiments being the first phase to evaluate the suitability of the models in the selected domain; all the metrics are reviewed without specification of the confidence interval. Area under curve (AUC) also will be included as a metric for evaluation in the next set of experiments.

RETRACTED

## 9. Key Constructs of Security Knowledge Management System

As part of building a knowledge system that takes in data and creates valuable information, some of the critical properties to be accounted for are discussed here. As part of BERT, labeling the training data and tokenization results in loss of traceability of the original word and the token. As the answer to the question is explored, it is crucial to figure out the position of these words that form the response from the context statement. One of the approaches would be to identify the answer string with a unique identifier that can be easily identified from various identifiers. TensorFlow and PyTorch being the approaches available, for application of transformers, Hugging Face provides the PyTorch interface. Pytorch sticks to API (ppplication programming interface) provision, not worrying about the internal workings of the approach, whereas TensorFlow provides insight into the inner workings of the approach, but that may sidetrack from the primary intention of this approach. The distinction between the workings of TensorFlow and PyTorch is made based on the earlier experience of working with PyTorch. BERT also provides various classes that intend to perform different tasks like token classification, question answering, next sentence prediction, and so on. Choosing the maximum length of the sequence is critical to the trade-off for the computational expense involved. If the maximum length is 512, it takes 4x longer to train than the length of 256 and 16x more time for 128. Hugging Face has used 384 lengths for the sequence in its implementation.

Truncation of the sequence results in a loss of answers for some of the questions. This is because, generally, answers are the last part of the sequence of sentences. In case if sentences are cut off during truncation, there is a higher possibility of losing the answers for some of the questions.

One possible way to handle this would be to truncate the context sequence from the beginning instead of the end. This truncation would involve significant effort, and it needs to be traded off for the returns from this. One of the ways would be to skip the questions where the context was truncated. Ninety-seven training examples were lost due to truncation from among 87,502 samples of the SQuAD. Fine-tuning of the BERT model involves predicting a category to call out if the token is identified correctly for the start of the span and another for the end of the span. Fine-tuning of the model is an attempt to increase the expertise of the model from being good at the text to the capability of question answering.

## 10. Learning from Source Code

In [54], the authors proposed an adaptive deep code search method for training once and then reusing the same in new code bases. This approach optimizes the need for training the codebases every time for search purposes. Though there are many programming data available in online sources like Stack Overflow, there is a lack of sound natural language processing-related approaches to extract code tokens and software-related named entities. In [55], the named entity recognition approach is proposed on code for named entity recognition. In [56], there is an exploration of topic modeling to mine unstructured software engineering data. This work surveyed topic modeling applications and identified an increasing need to focus on tasks associated with comprehension of source code and software history. In [57], code flaws and vulnerabilities modeling are focused on using the deep learning-based long short-term memory model, focusing on learning semantic and syntactic features of the code. In [58], a systematic literature review for multilanguage source code analysis is presented. This study helps explore the focus areas for development like static source code analysis, refactoring, detection of cross-language links, and other vital areas. In this study, statistical modeling of the source code is one of the focus areas. This statistical learning and representation of the source code can be based on these applications like static source code analysis, refactoring, and detection of cross-language links. Here, cross-language means multiple software programming languages. Language modeling study will be leveraged to model the natural language-related data that gets accumulated during the process of software development. And source code itself has naturalness in it which is more structured compared to the natural language text. This provides further opportunities for modeling the source code.

RETRACTED

In the software development landscape, software source code forms a critical component that potentially holds quite a pattern that can provide insight into potential software security vulnerabilities that can creep into the system. Devising a mechanism to model source code will add to the intelligence built via a software security knowledge management system. The idea would be to derive the pattern hidden in the program by modeling the property of the code. Code2vec is the recent popular approach that attempts to learn the distribution representation of the code. The thought process is detailed in [59], where authors try to present a neural model where the code is represented as a continuous distribution of vectors. This approach will help model inherent semantics property that is at the core of code semantics. Code is in the form of a collection of paths that is part of abstract syntax tree representation. Method name prediction is attempted in this work consuming the vector representation of the body. Twelve million methods of code are used as input for this modeling. In this approach, code snippets provide information to be represented as a bag of context, and a vector representing the context, the value of the same need to be learned. Work here revolves around finding a meaningful way to break up the code into smaller significant blocks and then aggregating these building blocks to arrive at meaningful predictions.  Figure 5 expresses the overview of the code2vec.

The general approach shows that a program needs to be taken in as input and broken into meaningful parts, converted to vectors that can then be aggregated into predictions. While the features are devised for this modeling approach, there is a trade-off between the effort involved for the model to learn and the effort involved in building those features. AST approach helps balance these factors by banking on the syntax associated with the code. AST paths are set as vectors here, which will include token vectors and path vectors. Tokens are the entities that are connected by the specific path in AST. All the tokens vectors and path vectors are combined as a matrix for which the tanh function is applied to bring in element-wise nonlinearity to rescale all the vectors between –1 and 1. A fully connected layer will provide a path context that encapsulates all the patterns in this part of the code sequence. The challenge would be to take in all the path contexts and aggregate the same into a code vector. There are three approaches to aggregate the path context: take the most crucial path context, take an average of all, and take the final one to bring attention and compute the weighted average of all the path context. As part of attention, vectors learn the semantic meaning of the path context and attention needed by the path context. The learned attention vector is the randomly initiated component that learns in parallel in the network. Path context vector and attention vector are combined with dot product to obtain scalar normalized with softmax to get the score that sums to one. Path context vectors are then multiplied by the normalized scalar values summed up to get the code vector. Code vector is the weighted average of the input vectors continuously learned and updated by the network during the learning phase. Target method name vectors are also trained with 14 million methods examples; these are used as a reference for validating the predictions done by the network.

In [60], the author proposes a neural source code representation with AST. The author here focuses on the fundamentals of extending code modeling for further analysis. Information retrieval methods would consider the code as text and miss the semantics understanding of the source code. ASTs are leveraged by the authors as the better approach to represent the code. ASTs, by nature, end up being long data sets way they represent the code. Instead of working on the entire ASTs, this proposed model works on split AST smaller statement trees.

RETRACTED

Furthermore, these are encoded into vectors, which will retain lexical and syntactic knowledge of statements. These statement vectors are modeled with bidirectional RNN, which will use the naturalness of these representations and help optimally represent the code in vector format. Authors have applied this model of code representation for solving code classification problems and code clone detection problems. Code classification approach will be explored to fit into the framework being explored here for smart requirements management. Authors have provided their implementation scripts in https://github.com/zhangj111/astnn.

The implementation proposed for the code classification will help model the code data and explore any vulnerabilities in the code. For this purpose, either training data can be built to train further this architecture of specific code data from the projects of the insurance company targeted for this security management framework for software development. Or implementation can be reused on local data as it is already trained on the C# language, the target language for this framework experimented with within this paper.

Implementation for code classification has a class written called pipeline that will parse the source code; split the data into training, developing, and testing; construct the dictionary; and train a word embedding. Further block sequences are generated for index representation, and data is processed for training purposes. Pipeline.py also uses the prepare_data.py for some of the functions. Further prepare_data.py uses class AST node from tree.py script. The class used here helps configure AST from the source code. In the train.py script, the author has configured a training approach. Model.py is referred to in the script train.py for running the model-related script. Train.py reads in train, test, and validation data runs the word2vec on the data and creates the embeddings. Parameters in Table 6 are configured for the model, BatchProgramClassifier.

The authors have reported an accuracy of 98.2% for the code classification task; this needs to be validated for the insurance company project data targeted for building the software security vulnerability modeling framework.

## 11. Conclusion

This paper has explored various building blocks that can be helpful build a comprehensive vulnerabilities management system for software development processes. The security of the software systems is the topmost priority for the software organization. Therefore, it is essential to leverage all the information generated across the industry and within the company. Various data science methods have been explored to build a knowledge management system that can assist the software development team to ensure a secure software system is being developed. Various approaches in this context have been explored using data of insurance domain-based software development. These approaches could facilitate an easy understanding of the practical challenges associated with actual-world implementation. The capabilities of language modeling and their role in the knowledge system were also discussed. The source code has been modeled to build a deep software security analysis model. The proposed model can help software engineers build secure software by assessing the software security during software development time. Extensive experiments have been drawn by considering the various machine learning and deep learning models. It has been observed that the proposed deep learning-based models can efficiently explore the software language modeling capabilities to classify software systems' security vulnerabilities. Distill BERT and BERT have shown the good capability to model the insurance domain data to learn the security loopholes in the software development processes. Experiments also have demonstrated the capability of attention models in software security modeling.

RETRACTED

## Figures and Tables

**Figure 1:** Working of sentence encoding.

**Figure 2:** BERT architecture.

**Figure 3:** Software security model architecture.

**Figure 4:** Input sequence illustration in BERT.

**Figure 5:** Overview of the code2vec.

**Algorithm 1:** Text classification using CNN.

**Algorithm 2:** Classification using bidirectional LSTM and attention layer.

**Algorithm 3:** Classification using USE with TensorFlow 1.0.

**Algorithm 4:** Neural network language model.

**Algorithm 5:** BERT for tokenization and feature creation.

**Algorithm 6:** DistilBERT for tokenization.

**Algorithm 7:** BERT with DCNN model.

**Algorithm 8:** SQuAD dataset process.

**Table 1:** DCNN architecture training specification.

Parameter	Value
Vocabulary size	Based on the vocabulary size of the tokenizer
Embedding dimension	200
Number of filters	100
Feedforward network units	256
Number of classes	2
Dropout rate	0.2
Epochs	1
Training	False

**Table 2:** DCNN model construct.

Layer	Configuration
Embedding	Vocabulary size, embedding dimension
Convolutional 1D bigram	Kernel size = 2; padding = valid; activation = ReLU
Convolutional 1D trigram	Kernel size = 3; padding = valid; activation = ReLU
Convolutional 1D fourgram	Kernel size = 4; padding = valid; activation = ReLU
Pooling	GlobalMaxPool1D
Dense	Activation = ReLU
Dropout	0.2
Last dense (for 2 classes)	Units = 1; activation = sigmoid
Last dense (for more than 2 classes)	Units = number of classes; activation = softmax
Loss (for 2 classes)	Binary cross-entropy
Loss (for multiclass)	Sparse categorical cross-entropy

RETRACTED

**Table 3:** BERT question answering system library specifications.

Modules	Library
Tensorflow	Tensorflow hub
official.nlp.bert.tokenization	FullTokenizer
official.nlp.bert.input_pipeline	create_squad_dataset
official.nlp.data.squad_lib	generate_tf_record_from_json_file
official.nlp	Optimization
official.nlp.data.squad_lib	read_squad_examples
official.nlp.data.squad_lib	FeatureWriter
official.nlp.data.squad_lib	convert_examples_to_features
official.nlp.data.squad_lib	write_predictions

**Table 4:** BERT question answering system training phase specifications.

Parameter	Value
Training data size	88 641
Number of training batches	500
Batch size	1
Number of epochs	1
Initialized learning rate	5*e* − 5
Warmup steps	10% of the number of training batches

**Table 5:** Comparison of all the experiments.

Experiment	Process	Output
CNN and FastText embedding	CNN-based processing	Accuracy: 71.89%; precision: 0.88; recall: 0.72; F1-score: 0.77
Bidirectional LSTM with FastText embedding	Bidirectional GRU or LSTM with global attention	Accuracy: 84.33%; precision: 0.91; recall: 0.84; F1-score: 0.87
USE model	USE pretrained model with TF 1.0	Accuracy: 92.61%; precision: 0.95; recall: 0.93; F1-score: 0.93
NNLM	NNLM-based sentence encoder, with pretrained model	Accuracy: 90.16%; precision: 0.81; recall: 0.90; F1-score: 0.86
BERT	BERT tokenization and TF Keras modeling	Accuracy: 91.39%; precision: 0.92; recall: 0.91; F1-score: 0.88
DistilBERT	DistilBERT-based preprocessing of data	Accuracy: 94.77%; precision: 0.95; recall: 0.95; F1-score: 0.94
BERT	Data preprocessing and tokenization with BERT	Accuracy: 97.44%

**Table 6:** Model configuration for BatchProgramClassifier.

Parameter	Value
Hidden dimension	100
Encoding dimension	128
Labels	104
Epochs	15
Batch size	64
Maximum tokens	Based on word2vec embeddings
Embedding dimension	Based on word2vec embeddings

## Data Availability

The data used to support the findings of this study are available from the corresponding author upon request.
